The article "Aortic Blunt Trauma Analysis during a Frontal Impact" was published in 2021. Journal: Appl Bionics Biomech.

# Aortic Blunt Trauma Analysis during a Frontal Impact

**DOI:** 10.1155/2021/5555218

**Published:** 2021-07-19

**Authors:** Mario Alberto Grave-Capistrán, Arturo Yishai Prieto-Vázquez, Christopher René Torres-SanMiguel

**Affiliations:** Instituto Politécnico Nacional, Escuela Superior de Ingeniería Mecánica y Eléctrica, Sección de Estudios de Posgrado e Investigación Unidad Zacatenco, 07738, Mexico

## Abstract

The aorta is the largest artery of the human body, and it is considered in the continuous medium mechanics as a hyperelastic material for its biological properties. The thoracic aorta is directly affected in vehicular collision events by compression generated between the ribcage and the three-point seatbelt tension producing injuries in the artery wall. A three-dimensional model of the thoracic aorta was constructed from digital tomographic images considering the ascending aorta, the aortic arch, and the descending aorta. The model obtained presents acceptable characteristics such as a length of 222.8 mm and an ascending aortic diameter of 22.7 mm, 22.7 mm in the aortic arch, and 16.09 mm in the descending aorta. A 150 ms time numerical simulation was developed through the finite element method (MEF), and the model was analyzed simulating a compression load on the artery at its front location. Boundary conditions were considered by selecting specific nodes in the model, such as the points where the artery is held in the thorax with other elements. In addition, displacement nodes were considered to establish a natural behavior of the artery. The outcomes show significant displacements in the artery wall. The most affected areas are the aortic arch and descending aorta, whose displacements reach 14 mm from their original position. Based on the abbreviated injury scale (AIS), the degree of injury to the aorta in this collision event is estimated, an AIS 2 with a moderate severity index and required medical attention.

## 1. Introduction

Traffic accidents are considered scenarios in which the human body can suffer several traumas. Three-point retention systems prevent the head and thorax from impacting the dash and steering wheel, causing injuries on the rib cage due to the compression effect between the seat belt and thorax. The aorta is one of the affected arteries structurally, harming the aortic wall. Aortic trauma is a life-threatening event characterized by fatal injuries such as lacerations and tears in the aorta. Blunt trauma spontaneously interrupts the circulation of the human body blood flow to the vital organs, affecting the victim's life. The worst situation causes immediate death, and traffic accidents are the leading cause of this trauma. Compression injuries to the thoracic aorta are generally in the aortic arch and descending aorta. Forceful cardiac rupture occurs more frequently in traffic accident events (73%), and cardiac injury has a mortality rate of 89%. 98% of the victims involved in car accidents with aortic injuries are classified in AIS3, and most of them died at the scene accident. The literature reports that the aortic arch suffers a critical injury, and 95% of victims with an aortic rupture undergo immediate surgical intervention survive [1–4]. Statistics about injuries on the chest in crash scenarios have been made by analyzing the most common injuries by wearing a seat belt. Percentages were established for a fatal aortic injury; the United Kingdom with 98.10% and the United States of America with 91% in frontal car collisions using a seatbelt. Although the seat belt reduces the risk of traumatic injuries in the body, there is a possibility of blunt trauma in the organs after a high impact which transfers energy directly to the thorax affecting the thoracic aorta. The study indicates a high percentage of aortic injuries using the seatbelt in a frontal collision. Although the airbag is activated, chest injuries are still serious to the internal organs. The traumatic injuries occur in the arms and pelvic area, and bruises are also generated through the chest and abdomen. The arteriograms confirm that there are traumatic injuries in the thoracic aorta, mainly in the descending aorta, it was determined that the harm was caused by the compression of the two-point or three-point seat belt, associating them with the “seatbelt syndrome” [5, 6]. Studies have been carried out on thoracic trauma and aortic rupture in frontal collision traffic accidents. The energy required to compress a soft tissue is proportional to the stress applied and material deflection. It has been established that the organs are described as viscous material characteristics, and the compressive force is proportional to the impact speed. In a certain amount of energy, when the impact speed rises, the consequence is that chest compression tolerance decreases. It has been confirmed by experimental evaluations of the theories about frontal and lateral impacts in high-speed events (more than 33 km/hr). In addition, high-speed situations produced injuries in the thoracic internal organs which are critical, particularly heart ruptures such as the thoracic aorta and large vessels of the circulatory system [7]. The aorta has been evaluated in its parts (ascending aorta, aortic arch, and descending aorta) considering that there is a joint to the thoracic spine, the heart, and the supra-aortic trunks, and it is estimated that the causes of the rupture of the artery are a sudden displacement of blood flow towards the aortic isthmus (hammer blood), a compression of the bony artery structure of the rib cage with the thoracic spine, and the effect of tension-torsion due to a sudden deceleration [8].

The article "Aortic Blunt Trauma Analysis during a Frontal Impact" was published in 2021. Journal: Appl Bionics Biomech.

On the other hand, numerical simulations have been developed involving the behavior of the thoracic aorta when it is subjected to compression loads, simulating both lateral and frontal vehicular collision events. Demiray and Holzapfel developed numerical simulations applying mathematical tensors to represent the aorta mechanical properties. Boundary conditions are considered in specific parts of the artery (the aortic arch, supra-aortic trunks, and descending aorta). Tension in the artery is generated, severely injuring the ascending aorta [9]. The Wayne State Human Body Model (WSHBM) is a computational tool that integrates somebody's region such as the shoulders, ribs, and thorax, and it has been found that the maximum principal stresses after applying stress to the aorta are between 102 kPa and 136 kPa [10]. With LS-DYNA software, the aorta was considered as a transversely isotropic element of an incomprehensible hyperelastic material. It has been found that in a left lateral collision at a speed of 27.6 km h-1 in a time of 90 ms, the Von Mises stress peak is 1.8 MPa [11]. The following mechanical properties were assigned considering the aorta as an elastic material: density of 1.20 E-06, Young's modulus of 5.00 E-03, and Poisson's ratio of 0.40. Results reveal that the descending aorta presents a maximum peak value of 0.148 kPa. On the other hand, the maximum value obtained for the aortic bulb was 0.263 kPa, and the maximum value of stress was 55.4 kPa.

These values are interpreted as serious in specific artery areas such as the aortic arch [12]. The methodology for the three-dimensional modeling of parts of the human body is considered important; studies on compression loads with an average acceleration of 6.51 in the human thorax were performed, and it has been found that a compression load of 5.16 N generates a deflection in the rib cage of the human body causing injuries to internal organs. The rib cage is one area in the human body that suffers injuries due to car accidents or high-energy traumas. Studies report that injuries to the thorax can be fatal in a car accident. Studies conducted on the chest's behavior in different load scenarios show that the energy generated by the automotive impact is transmitted to the organs inside the rib cage. Analyses were performed on lesions in the thorax using a six-year-old Hybrid III finite element model. Applying standards based on the evaluation of rollover car crashes; it was recorded that the thorax of the human body gets more damage when a seat belt 3 points is used, and the deflection in the chest reaches up to 6.21 mm. Applying the Chest Severity Index using a finite element model Hybrid III dummy type in a frontal car collision, lesions in the thorax with a high degree of mortality are reported. Numerical simulations of 120 ms period time have been created, and the lesions in the thorax have been analyzed in frontal crash tests, boundary conditions are considered and are automatically assigned by the software, passive safety elements such as the seat belt generates compression loads that cause injuries to the rib cage [13–16]. Finally, a viscoelastic fractional model applying MEF has been used to create numerical simulations dividing the artery wall into its 3 layers: the intima, the media, and the adventitia. The layer's behavior determines the distribution of stresses and the deformation in the artery under the Von Mises criteria [17].

The article "Aortic Blunt Trauma Analysis during a Frontal Impact" was published in 2021. Journal: Appl Bionics Biomech.

This research is aimed at analyzing the structural behavior of the aorta by a numerical simulation in different compression steps due to frontal crashes. Furthermore, the results focus on establishing a relationship with the type of injury and structural damage working as a predicting damage method of the thoracic artery. In addition, the present study goes further than the available literature on the aortic wall analysis through the construction of a numerical simulation based on programmable control instructions solved by specialized mathematical language and using the FEM applied to three-dimensional modeling obtained from TC. Thus, results show a perspective of the structural behavior of the aorta in different compression steps due to frontal impacts in a car, highlighting substantial displacements in the artery wall.

## 2. Materials and Methods

Following the proposed methodology presented in Figure 1, a detailed model was developed with the literature's characteristics and will allow it to be subjected to numerical simulations applying FEM. The thoracic aorta's three-dimensional model began by identifying the parts and the specific location within the human body. The research was carried out based on clinical and biological reports. A computer program that allows artery reconstruction was also selected to develop a three-dimensional model. The parts were evaluated from a preliminary model with the characteristics to be subjected to numerical analysis.

Based on the literature on the artery's biomechanics and the clinical reports collected for this research, it is determined that the aorta receives compression stress from the tension generated by the three fastening points that the seatbelt integrates into a car. The inertial force of the frontal impact forces the human body to move forward with an inclination towards the car's steering wheel. The seat belt is activated, retaining the human body avoiding an impact with the dashboard, awning, or steering wheel. From this event, the compression stress is generated towards the thorax, initially affecting the bone structure of the rib cage and, in particular, the sternum, the stress transmission towards the internal organs of the human body, such as the thymus and the aorta.  Figure 2 represents the frontal collision event and the parts of the human body affected by the retention of the seat belt (sternum, thymus, and aorta).

The article "Aortic Blunt Trauma Analysis during a Frontal Impact" was published in 2021. Journal: Appl Bionics Biomech.

### 2.1. Three-Dimensional Modeling of the Aorta

The three-dimensional modeling of the thoracic aorta was developed through the SCANIP® computer program. First, the artery was reconstructed from a sequence of 222 digital images belonging to the thorax of the human body of a 50th percentile Mexican patient. The best way to obtain a three-dimensional model is through computed tomography (CT). Therefore, these digital images were configured as a complete data range in order to obtain the best resolution in each image. In addition, a mask was configured to identify the parts of the thoracic aorta, and through the work interface of the computer program divided into the three cross-sections it uses (horizontal, sagittal, and frontal), the three-dimensional model reconstruction of the thoracic aorta contemplates the geometry based on clinical reports.

The reconstruction process identifies the specific areas of the thorax in which the thoracic aorta is located. The mask created has the purpose of indicating the parts of interest of the model to be generated (ascending aorta, aortic arch, and descending aorta). Also, the artery elements are considered boundary conditions, as fixation points were considered: the aortic bulb and the supra-aortic trunks (brachiocephalic trunk, left common carotid artery, and subclavian artery). The cleaning process of the digital images was carried out by preserving the pixels that make up the thoracic aorta in each layer. The model generated in SCANIP® is a three-dimensional solid body, and a Gaussian filter was applied to erase roughness on the surface of the three-dimensional model to be used in any other computer program.  Figure 3 shows the three-dimensional model of the thoracic aorta. The geometric dimensions are indicated in each of the parts of the artery.

### 2.2. Numerical Requirements

The Meshmixer® software provides tools to repair the 3D model obtained from SCANIP®. First, the whole model was inspected and fixed; the artery wall thickness was specified based on the literature, with a tubular layer of 2.3 millimeters, and was configurated for the three parts of the aorta (ascending, aortic arch, and descending). In Figure 4 is observed a human aorta model for numerical simulation.

The article "Aortic Blunt Trauma Analysis during a Frontal Impact" was published in 2021. Journal: Appl Bionics Biomech.

In Meshmixer®, it is established in the surface boundary conditions in the aortic bulb and the supra-aortic trunks.  Figure 5 shows the flat faces created in the aortic arch corresponding to the ligamentum arteriosum and the anterior longitudinal ligament of the thoracic aorta located in the third vertebra and where the aorta is attached.

Once the anatomical characteristics of the aorta and the boundary conditions had been established, in a final stage, the complete model was created as a solid to avoid errors during the numerical simulation to obtain correct results. A file with STL characteristics was created to import to Matlab® software for numerical simulation.

High-energy traffic accidents in frontal collision scenarios are responsible for blunt trauma to the human body due to their impact on different parts. The purpose of using restraint systems (three-point seatbelt) is to avoid the most significant number of injuries to the passenger. However, when the impact is brutal, compression loads are generated between the thorax and the seat belt, causing injuries directly to the human aorta, producing from superficial signs such as ecchymosis in the chest to closed traumas in the aorta such as lacerations, aortic dissections, and ruptures that represent chronic complications to the victim and sometimes immediate death. The NCAP (New Car Assessment Program) is a European standard used in the automotive to evaluate motor vehicles' structural functionality and safety systems. The Latin-NCAP is the current regulation applying in Mexico. Its evaluation analyses frontal collision events against objects such as safety barriers, concrete structures, and other vehicles [18, 19].

For the construction of the numerical simulation, the standards and evaluation criteria of the Latin-NCAP are considered. The basic assessment configuration in safety systems proposed by the standard in frontal collision events in sedan-type cars with a mass between 1500 kg and 2000 kg is described below:

1. The frontal impact occurs at a speed of 64 km/h (40 m/h)
2. The vehicle hits an off-center barrier in the driver's position
3. The front of the barrier is deformable
4. The safety systems (3-point seatbelt, front and side airbags)

The standard considers that 40% of the frontal impacts the structure against another element in most traffic accidents. The vehicle's energy absorption is high in the impacted part (driver or front passenger), so injuries to the human body can be severe and fatal.  Figure 6 represents the frontal collision event standardized by Latin-NCAP [20].

The article "Aortic Blunt Trauma Analysis during a Frontal Impact" was published in 2021. Journal: Appl Bionics Biomech.

The Latin-NCAP evaluates the impacts in 150 ms, using the Abbreviated Injury Scale (AIS) to determine the injury in the human body. In most of the passengers, the chest protection is adequate during a frontal impact. However, critical injuries in internal organs such as the aorta that can be affected are not ruled out.

The numerical simulation is focused on the displacements generated in the three-dimensional model when stress compression occurs. It also contemplates the inertial action acquired by the frontal impact and the compression stress generated in the thorax by the seatbelt, which transmits payloads to the ascending aorta of the human body. The artery model is considered hyperelastic material in the geometric structure, bringing the numerical simulation to real conditions and verifying the proposal under the standards by the regulation considered. The three-dimensional model is in a vertical position, the loads are applied to the back of the 3D model (descending aorta) as an effect of the inertial movement of the frontal impact and in the frontal part (ascending aorta) due to the compression exerted by the three-point seatbelt, and Figure 7 shows the assigned forces on the “*y*” axis.

Mechanical properties were assigned considering the Ogden constitutive model.  Table 1 shows the values for the structural configuration of the aorta model [21, 22].

### 2.3. Methodology for the Numerical Analysis

Matlab® software was used to import the STL, and through an open-source computer program, the preprocessing and postprocessing were structured. The STL file was load with specific commands, preserving the original model without disturbing the geometry and structure. This computer program allows the user to establish criteria on the model that allow it to be adapted to carry out numerical simulations in different circumstances. Initially, the general configuration was established through instructions based on C languages, such as font size, label location, and the three-dimensional model's visual field. Once the preliminary configuration was completed, the model was imported, instructions were established to specify the origin of the file, and finally, Matlab® shows it in the default graphical interface. Thus, the model preserves the original geometry established in the previous packages. Hence, it should be noted that the three axes' dimensions are those obtained from the 3D model built-in SCAN IP®.  Figure 8 shows the 3D model of the aorta with the assigned characteristics.

The article "Aortic Blunt Trauma Analysis during a Frontal Impact" was published in 2021. Journal: Appl Bionics Biomech.

The numerical simulation will perform in the region for the 3D model. The generated code analyses the input elements in the imported model and transforms them into tetrahedral finite elements. The imported model contains an internal conduit that also acquires the same mesh.  Table 2 shows the values of the assigned mesh to the imported 3D model.

The model is completely mapped in the finite elements selected for the structural analysis. The size of each of these tetrahedral elements is adequate concerning the computational resource required to build the numerical simulation. The finite elements created are shown in Figure 9, a close-up image, the facets of the tetrahedral elements are appreciated.

Based on the human body's anatomy and chest, specific boundary conditions are contemplated in the three-dimensional model, such as the ascending aorta, the aortic arch, and the descending aorta selected by control structures code created on the faces and nodes the model's surface. Each node's location contains a specific value for each of the axes, including negative values that are part of the imported three-dimensional model space. Matlab® software interprets the entire model in a three-dimensional space in which each point in the model has a specific coordinate and the size of the finite element. The selection of the boundary conditions was through commands and logical operators that allowed the points and nodes' location within the three-dimensional model. In the reconstruction of the 3D model of the aorta, the final part of the aortic bulb was considered a flat face to adapt and obtain the selection of corresponding nodes. The aortic arch is the following part of the thoracic aorta; it joins the ascending aorta and the descending aorta. In addition, on the crest of the aortic arch, there are the supra-aortic trunks distributed towards the arms of the human body and the right and left frontal lobes of the brain. The boundary condition zones in the aortic arch were considered based on literature. The support nodes were attached in the same way as in the ascending aorta, and the mapping was carried out in this area and the nodes corresponding to the points considered. The aortic arch section presents the most significant number of nodes selected for the boundary conditions, adapting to the conditions involved in the human body anatomy. The last part of the thoracic aorta is the descending aorta. It acquires this name since it is directed towards the lower part of the human body. In this particular area, the end of the three-dimensional modeling is considered a boundary condition, as in the ascending aorta, a flat face was adapted at the end of the duct to achieve the mapping identification of the node's coordinates. Furthermore, since the case study only involves the thoracic aorta, it was decided to close the duct of the descending aorta without affecting the geometry; most of the nodes of movement (blue ones) are found in this section of the aorta, between the aortic arch and the descending aorta.

The article "Aortic Blunt Trauma Analysis during a Frontal Impact" was published in 2021. Journal: Appl Bionics Biomech.

On the other hand, movement faces and nodes in the model also represent a fundamental function for developing the numerical simulation. During frontal vehicular collision events, the human body suffers a forward displacement due to deceleration. The safety restraints prevent the impact of the thorax and head with the car's internal elements but generate compression loads on the rib cage. The aorta undergoes compression stress that displaces the aorta in its free parts and does not share contact, such as the boundary conditions described above. It is determined that the nodes in blue tonality without considering the designated boundary conditions assume the characteristic of movement in the three axes that involve the three-dimensional working space.  Figure 10 shows specific points to set the boundary conditions and the boundary conditions set.

Boundary condition points established in the model are very close and similar approximations compared to the literature. In addition, the settings integrated into the model must also be configured concerning the appropriate axis allowing to determine the points that should not be displaced when a load is presented. However, if it is of high magnitude, the clamping points are affected.

The FEBIO® solver with Matlab® was used to simulate compression in the frontal part of the 3D model. A color bar shows the displacements generated in the modeling; load simulation shows the displacements from the initial position and acquires shades concerning the color bar. In addition, the results are shown graphically as a function of the stress applied. The Cauchy stress is considered a function of time, and a graph of the displacements is generated in the model; the duration of the simulation (applied load) does not exceed 150 ms as established by the Latin-NCAP regulations.  Figure 11 shows the components of the numerical simulation.

The frontal collision focuses on evaluating the artery compression by seatbelt load generated by the restraint system. During the numerical simulation, results were obtained for the three specific parts of the aorta: ascending aorta, aortic arch, and descending aorta. The aortic bulb, the supra-aortic trunks, and the descending aorta are unable to move in the three three-dimensional axes. In comparison, the boundary conditions of the left pulmonary artery and the boundary condition in the posterior part of the model are assigned to disable the movement in the three axes. AIS classifies the injuries that are generated in the human body. It is divided into body region, type of anatomic structure and specific anatomic structure. The displacements, and type of injury in the elements of the rib cage (internal organs) are related to the AIS scale considering the type of injury generated in the aorta.  Table 3 shows the classification about the blunt trauma at the aorta according to AIS codes.

The article "Aortic Blunt Trauma Analysis during a Frontal Impact" was published in 2021. Journal: Appl Bionics Biomech.

Holzapfel's constitutive model is one of the most accepted models to describe arteries. It is a simplified model of the arterial wall in which it is assumed that the response is by two materials that make up the structure of the artery wall. This model is formulated based on the terms of the invariant, the function of the strain energy of the tension-based Cauchy and quasi-incompressible, obtaining the following expression:

(1) $$\begin{array}{c} W=\frac{\mu }{2}\left(I_{1}-3\right)+\frac{k_{1}}{2k_{2}}\underset{\propto =4,6}{\sum }\left[e^{k_{2}{\left(I_{\propto }-1\right)}^{2}}-1\right]. \end{array}$$

Furthermore, Holzapfel's viscoelasticity determines the energy density to infinite time can be described as follows:

(2) $$\begin{array}{c} W^{\infty }\left(C\right)=W_{\text{vol}}^{\infty }\left(J\right)+W_{\text{iso}}^{\infty }\left(\bar{C}\right). \end{array}$$

The function of energy density is determined from *C* and considering certain internal variables of deformation Γ_*a*_, *a* = 1, ,,*m*, as follows:

(3) $$\begin{array}{c} W=W\left(C,\Gamma_{1},,,\Gamma_{m}\right)=W_{vol}^{\infty }\left(J\right)+W_{iso}^{\infty }\left(\bar{C}\right)+\overset{m}{\underset{a=1}{\sum }}Y_{a}\left(\bar{C},\Gamma_{a}\right). \end{array}$$

Acquiring the following normalization conditions:

(4) $$\begin{array}{c} {\text{W}}_{\text{vol}}^{\infty }\left(1\right)=0,\\ {\text{W}}_{\text{iso}}^{\infty }\left(I\right)=0,\\ \overset{m}{\underset{a=1}{\sum }}Y_{a}\left(I,I\right)=0. \end{array}$$

Description through models for describing the mechanical behavior in order to obtain stress and strain patterns applied in organic tissues such as the human aorta. Ogden model is considered as an applicable model with hyperelastic material behavior and expresses the strain energy *W* considering the main extensions: *λ*_1_, *λ*_2_, *λ*_3_.

This mathematical model generates results with an acceptable approximation in stress tests. The applicable expression is

(5) $$\begin{array}{c} W=\overset{n}{\underset{p=1}{\sum }}\frac{u_{p}}{\alpha_{p}}∙\left(\lambda_{1}^{\alpha p}+\lambda_{1}^{\alpha p}+\lambda_{1}^{\alpha p}-3\right). \end{array}$$

The article "Aortic Blunt Trauma Analysis during a Frontal Impact" was published in 2021. Journal: Appl Bionics Biomech.

## 3. Results

During the execution of the numerical simulation, there are specific points in which the aorta's behavior is appreciated when compression stress is applied. For example, in the milliseconds of 24.90, 49.80, 74.70, 99.60, 124.50, and 149.40; it is possible to visualize the displacements in specific areas of the aorta from the aortic bulb to the descending aorta, and the behavior based on the mechanical properties and characteristics of the model is adequate considering the stress applied. Although the numerical simulation duration is 298.00 ms, the compression effect in the aorta ends at the instant of 149.40 ms, and total displacements in the artery are generated at this period.  Figure 12 presents the behavior of the aorta at the periods mentioned.

The artery displacements generated explicitly in the descending aorta between the aortic arch and the last part of the descending aorta model considered all boundary conditions. However, the movement on the plane *“x”* involves esophagus contact (thoracic part). Therefore, the behavior of the thoracic aorta is essential, highlighting that the aortic arch is the area in which the highest displacement is generated from its position, the displacement in 124.50 ms increases to 14 mm, and is considered important because it is where the compression stress is concentrated.

## 4. Discussions

The study carried out presents a static analysis simulation on the behavior of the arterial wall of the thoracic aorta using MEF. The three-dimensional model developed is configured considering the mechanical properties of hyperelastic soft tissue. In addition, the study considers the origin of blunt trauma by compression loads due to a car collision. However, elements such as the car, passenger compartment, and seat belt are not considered.

An interesting behavior is observed in the common carotid artery since, during compression of the thoracic aorta, the central supra-aortic trunk presents a minimum, and constant displacement through time simulation, which is 1 mm. The position is away from areas that undergo displacement in the thoracic aorta (ascending aorta and aortic arch). The left subclavian artery shows a linear increase from 3 mm to 13 mm of displacement due to its proximity to the aortic arch, while the brachiocephalic trunk presents a maximum displacement reaching 7 mm. The ascending aorta has a maximum displacement up to 6 mm at 149.40 ms*. A*lthough the displacement is minimal, it can be considered fatal in higher-speed collision scenarios. Nevertheless, the aorta area does not present serious injuries based on the numerical simulation. Finally, the descending aorta increases an average of 2 mm simultaneously with a total displacement of 14 mm.

The article "Aortic Blunt Trauma Analysis during a Frontal Impact" was published in 2021. Journal: Appl Bionics Biomech.

It should be noted that considering the numerical simulation constructed, the behavior of the tubular structure near the aortic arch is forced to move to the esophagus (thoracic area).  Figure 13 presents the relation of the results shown in Figure 12, and the most affected area at 149.40 ms is the aortic arch, which is considered the part of the aorta with the most probability of a rupture. It is also observed that the points where the boundary conditions are concentrated to sustain the model are respected and present minimal displacements as part of the behavior that exists within the rib cage.

The displacements in the arterial wall generated by the compression load during the numerical simulation represent deformations in the artery. The properties that characterize the aorta are of the hyperelastic and viscoelastic types. Although the artery's displacements in the event of a frontal collision are considerable, they do not represent a failure in the material of the artery, so it can be considered that the artery suffers a sudden displacement in the aortic arch that can severely affect blood flow.

During the thorax's impact due to the tension of the seatbelt, the aforementioned car safety systems and the rib cage are also involved. Initially, the element that receives the highest stress compression is the sternum, and it is considered that the transfer of energy towards the aorta is important in relation to the car's impact speed. For this case study, at 64 km/h, the artery undergoes displacements up to 14 mm in the aortic arch and the descending aorta forcing the artery and the left pulmonary ligament to displace. Finally, based on the AIS scale, the degree of injury in the aorta is classified. Therefore, the code corresponds to an AIS 2 with required medical attention and injuries which are reversible. Results show that the aorta is displaced 14 mm from its original position and moderately affected due to contusion in the rib cage. According to the aorta structural behavior in the numerical simulation, it can compare with clinical analysis by Lorenzo et al., which report that the main deformation is at the aortic arch. Wei et al. made a 27 km/h lateral impact simulation, which describes the same behavior at the aortic arch in less displacement due to the stress by the 27 km/h scenario. Zhengwei et al. show the same aortic arch and descending aorta behavior with *5* mm displacement in 30 ms simulation compression load. Finally, Belwadi et al.'s lateral collision simulation shows that the left subclavian artery is also injured by the stress compression followed by the descending aorta according to its fringe level.

The article "Aortic Blunt Trauma Analysis during a Frontal Impact" was published in 2021. Journal: Appl Bionics Biomech.

Thus AIS 2 is the code selected for the trauma in this study case as a moderate injury describing there are no affectations to the organs as the numerical results shown in Figure 12.  Table 4 shows the AIS coding and its description.

Developed numerical simulations allow analyzing the thoracic aorta's structural behavior in compression load events due to stress by the car seatbelt. The numerical simulation can also set compression stress in three-dimensional models considering boundary conditions to emulate collision scenarios. Numerical simulation construction through specialized computational code by FEM allows creating a three-dimensional workspace, importing an STL object, setting any finite element, assigning material properties, and solving a case study applying stress on the object to predict material behaviors. The aorta's behavior with the applied mechanical characteristics is similar, establishing that the area most affected during compression loads by retention systems is in the aortic arch. It should be noted that the numerical simulation of this work does not include elements that are part of the case study (seatbelt and car) due to the limitation provided by the computer programs used. However, the numerical simulation built by programmed instructions contributes to the construction of any scenario for simulation in organs of the human body.

## 5. Conclusions

In this work, a numerical simulation of the structural aorta behavior was carried out in a static field, applying compression loads in the ascending aorta of a 3D model, which TC developed. Compression load simulation in the artery was carried out considering the boundary conditions at specific parts of the aorta emulating the stress applied by the tension of the strap of the restraint system of a car. The use of mathematical models based on mechanical tensioners allows the numerical simulation construction to establish the type of material according to the family of soft tissues in which the arterial wall belongs. Ogden and Viscoelastic model application in the solution by matrix methods sets the behavior in the mechanics of the continuous medium of hyper-elastic materials. According to the mathematical applied models, displacements were analyzed through a matrix solver considering the collision event. The anatomical-based coding system by AIS score describes the severity of injuries. Numerical results show that the thoracic aorta at the aortic arch reaches 14 mm displacement and does not represent major injuries to the artery. However, according to the AIS score and medical reports, sudden stress at 64 km/h on the thorax requires medical attention as a protocol in collision scenarios. The results of the proposal for this work are compared with those of other authors and clinical reports.

The article "Aortic Blunt Trauma Analysis during a Frontal Impact" was published in 2021. Journal: Appl Bionics Biomech.

## Figures and Tables

**Figure 1:** Flow diagram for the three-dimensional modeling of the aorta.

**Figure 2:** Thoracic injuries by seat belt compression.

**Figure 3:** Aortic characteristics obtained from SCANIP®: (a) aortic bulb diameter (22.7 mm), (b) Aortic arch diameter (21.96 mm), (c) Aorta descending diameter (16.09 mm), and (d) 3D model of the aorta.

**Figure 4:** Human aorta 3D model. (a) Thickness assignation to the model of the aorta. (b) Ascending aorta and descending aorta cuts.

**Figure 5:** Lateral and posterior aortic arch boundary conditions. (a) Flat face for the arterial ligament of the pulmonary artery and (b) flat face for the anterior longitudinal ligament of the thoracic spine.

**Figure 6:** Frontal impact against deformable element structure from Satué-Vallvé.

**Figure 7:** Forces application areas at the three-dimensional model parts.

**Figure 8:** STL model imported to Matlab®.

**Figure 9:** Three-dimensional model of the thoracic aorta in tetrahedral second-order finite elements.

**Figure 10:** (a) Dimensional model in (b) boundary conditions set.

**Figure 11:** Numerical simulation elements.

**Figure 12:** Aorta behavior by compression in milliseconds periods, 24.90, 49.80, 74.70, 99.60, 124.50, and 149.40.

**Figure 13:** Displacement-time graph of the thoracic aorta artery.

**Table 1:** Mechanical properties of the thoracic aorta.

Mechanical properties of the arterial wall of the aorta	
Young's modulus (*E*)	1000 kPa
Density (*ρ*)	1.2*e*^−6^ kg/mm^3^
Poisson's ratio (*γ*)	0.45
Shear modulus (*G*)	137 ± 18 kPa

**Table 2:** Elements for construction of the tetrahedral mesh in the 3D model of the thoracic aorta.

Mesh element	Number of elements
Points	1310
Tetrahedral	4118
Faces	9518
Faces on the outer limit	2564
Faces on the input facets	2564
Edges on input segments	3846
Steiner points within the domain	26

**Table 3:** AIS code and zones for the analysis of lesion in the thoracic aorta.

	AIS code	Zone
Body region	04	Chest
Type of anatomic structure	02	Blood vessels
Specific anatomic structure		
Type of injury	04	Contusion
Head-loss of consciousness (LOC)	N/A	N/A
Spine	04	Thoracic
Vessels, nerves, organs, bones, joints	02	Blood vessels

**Table 4:** AIS coding system.

AIS score	Injury	Description
0	None	None
1	Minor	Superficial
2	Moderate	Reversible injuries; required medical attention
3	Serious	Reversible injuries: hospitalization required
4	Severe	Life-threatening; not fully recoverable without care
5	Critical	Irreversible injury; not fully recoverable even with medical care
6	Unsurvivable	Deadly

The article "Aortic Blunt Trauma Analysis during a Frontal Impact" was published in 2021. Journal: Appl Bionics Biomech.

## Data Availability

The data used to support the findings of this study are available from the corresponding author upon request.
